# Tidal Volume Level Estimation Using Respiratory Sounds

**DOI:** 10.1155/2023/4994668

**Published:** 2023-02-16

**Authors:** Lurui Wang, Zhongwei Jiang

**Affiliations:** Graduate School of Science and Engineering, Yamaguchi University, Yamaguchi, Japan

## Abstract

Respiratory sounds have been used as a noninvasive and convenient method to estimate respiratory flow and tidal volume. However, current methods need calibration, making them difficult to use in a home environment. A respiratory sound analysis method is proposed to estimate tidal volume levels during sleep qualitatively. Respiratory sounds are filtered and segmented into one-minute clips, all clips are clustered into three categories: normal breathing/snoring/uncertain with agglomerative hierarchical clustering (AHC). Formant parameters are extracted to classify snoring clips into simple snoring and obstructive snoring with the *K*-means algorithm. For simple snoring clips, the tidal volume level is calculated based on snoring last time. For obstructive snoring clips, the tidal volume level is calculated by the maximum breathing pause interval. The performance of the proposed method is evaluated on an open dataset, PSG-Audio, in which full-night polysomnography (PSG) and tracheal sound were recorded simultaneously. The calculated tidal volume levels are compared with the corresponding lowest nocturnal oxygen saturation (LoO_2_) data. Experiments show that the proposed method calculates tidal volume levels with high accuracy and robustness.

## 1. Introduction

Sleep quality and sleep time are both important for human health. Sleep quality is the measurement of how restful and restorative the sleep process proceeds. Enough sleep hours do not necessarily guarantee to get the most restful type of sleep. More than 80 sleep disorders are known to affect sleep quality. Among all these factors that cause poor sleep quality, sleep-related breathing disorders (SRBD) is the second one of all sleep-related disorders (the first one is insomnia) [1]. SRBD is the condition of abnormal and difficult respiration during sleep, which has effects on the balance of oxygen and carbon dioxide in the blood. Tidal volume is one of the parameters for monitoring respiratory ventilation and pulmonary function. Tidal volume is the amount of air that moves in or out of the lungs with each respiratory cycle. The normal tidal volume is around 500 mL in an average healthy adult male and approximately 400 mL in a healthy female. The tidal volume during sleep can be measured by many methods, such as polysomnography (PSG) and inductance plethysmography [2]. However, these methods are expensive, require a specialized operation, and cause uncomfortable sleeping. Therefore, there is a need for a nonintrusive, easy-operating method that can be used in a home environment. The acoustic method is getting popular in respiration monitoring as it only involves acquiring and processing respiratory sound signals to estimate tidal volume. The development of smartphones and wearable devices also made it possible to monitor respiration and tidal volume during sleep. Monitoring respiratory quality using respiratory sound is becoming a hotspot in recent years.

Many researchers have focused on analyzing the correlation between respiratory sound and respiratory airflow due to its potential for assessing snoring risk and estimating tidal volume. Various models or algorithms are proposed to estimate respiratory flow through respiratory sounds. Gavriely and Cugell proposed that the breath-sound amplitude (BAS) and flow (*F*) generally follow a 1.75-power relationship [3]. Yap and Moussavi proposed a method to use average power and an exponential model to estimate respiratory flow through tracheal sound, which reached an estimation error of 5.8 ± 3.0% [4]. Reljin et al. used the blanket fractal dimension (BFD) as the parameter for estimating the tidal volume from tracheal sounds recorded by an Android smartphone, the smallest normalized root-mean-squared error of 15.877% ± 9.246% was obtained with the BFD and exponential model [5]. Yadollahi and Moussavi extracted the average power, the logarithm of the variance, and the logarithm of the envelope of tracheal sound as a feature, they compared the ability of these features to fit the flow-sound relationship, suggesting that the logarithm of the variance is the best feature to describe the flow-sound relationship with a linear model [6]. Other studies indicated that the Shannon entropy and sound variance also have an exponential relationship with the respiratory flow [7, 8]. Most of these papers indicate that the flow rate and respiratory sound amplitude follow a power law. This relationship used to estimate the respiratory flow rate can be presented in the following equation:

(1) $$\begin{array}{c} \log F_{est}=C_{1}\log\left(E\right)+C_{2}\text{.} \end{array}$$

*F*_est_ is the estimated flow rate (L/min), *E* is the respiratory sound amplitude, and *C*_1_ and *C*_2_ are the coefficients. *C*_1_ and *C*_2_ are determined by the human upper airway structure and can be calculated via a few breaths with a known flow rate for each participant, this procedure is called calibration. Current methods require calibration to determine the model coefficients *C*_1_ and *C*_2_. Yadollahi and Moussavi found that the parameters of the flow-sound relationship during sleep and wakefulness are different [9]. Therefore, for monitoring the tidal volume during sleep, the model parameters should be calibrated with sleep respiratory sounds.

However, these methods mentioned above are only applied to normal respiration, and calibration is needed for each case. Furthermore, these methods had not worked well for respiration during snoring. During snoring, the sound amplitude is higher than normal breathing, on contrary, the respiratory airflow is lower than normal breathing. The main reason is that the upper airway is usually collapsed or obstructed, and is highly variable during snoring. Respiration monitoring during snoring is important as it greatly affects sleep quality. During snoring, the upper airway is partially or completely blocked, and the respiratory airflow is limited or vanishes. Snoring usually leads to intermittent hypoxemia (IH), hypercapnia, arousal, hypertension, and sleep fragmentation. In this paper, a qualitative tidal volume estimation by a respiratory sound signal is proposed. It only used respiratory sound for analysis and does not need calibration. Therefore, the respiratory sound data could be easily collected by recording equipment and could be used in a home environment.

The proposed method consists of 4 main steps. First, the respiratory sounds are preprocessed into clips. Second, all clips are clustered into the normal breathing/snoring/uncertain categories with agglomerative hierarchical clustering (AHC). Third, the snoring clips are classified into simple snoring and apneic snoring with the *K*-means algorithm based on formant parameters and time domain parameters. Finally, the maximum breathing pause interval (MBPI) is calculated for apneic snoring clips to set the tidal volume to a medium or low level. The last time is calculated for simple snoring to set the tidal volume to a high- or medium-level. All the predictions are compared with LoO_2_ (lowest nocturnal oxygen saturation) to evaluate the performance. All steps are unsupervised and do not need any calibration. The flow of the proposed method is shown in Figure 1.

## 2. Materials and Methods

The tracheal sounds are extracted from the PSG-Audio dataset. The dataset comprises 212 polysomnograms along with synchronized tracheal sound. The dataset contains edf files comprising polysomnogram signals and rml files containing all annotations by the medical team [10]. The edf files contain 20 channels, the SpO_2_ (blood oxygen saturation level, in channel 15) and tracheal sound (in channel 19) data are extracted from the edf files for analysis. The SpO_2_ measures the amount of oxygen in the blood. The corresponding respiratory events (obstructive apnea/mixed apnea/hypopnea) are extracted from the rml files. The sampling frequency of SpO_2_ and tracheal sound is 1 Hz and 48000 Hz, respectively. A five minutes data clip is shown in Figure 2.

### 2.1. Agglomerative Hierarchical Clustering

#### 2.1.1. Processing

The first step of preprocessing is filtering and denoising. As the respiratory sound energy of healthy people is usually concentrated in the low-frequency range of [50, 2500] Hz, a 50–2500 Hz Butterworth bandpass filter is used to filter noise. The sampling rate of recording files is downsampled to 5000 Hz. The second step of preprocessing is segmentation. The duration of the clip length is settled by considering the micro and the macro aspect. One clip should be short enough to separate each breathing stage; therefore, the audio signal in one clip is stable. The length of the clip is better to be cut with 5 to 10 breath periods for analysis. The usual breath period during sleep is 3 to 6 seconds. The length of 30 seconds to 60 seconds is considerable. Furthermore, considering the time of apnea in a serious case, it usually takes more than 30 seconds. In this paper, the length of segmentation is set at 60 seconds.

#### 2.1.2. Feature Extraction

According to research about the human hearing mechanism, the human ear has different hearing sensitivity to sound waves of different frequencies. The human ear has a higher resolution of low-frequency sounds than high-frequency sounds. The Mel scale is a mapping from the human auditory perceived frequency to the actual frequency of the sound. By converting the frequencies to the Mel scale, features can better match the human auditory perception [6]. The Mel scale describes the nonlinear characteristics of the human ear frequency, and its relationship with frequency can be approximated by the following equation.

(2) $$\begin{array}{c} Mel\left(f\right)=2595*\;\log_{10}\;\left(\frac{f}{700}+1\right)\text{,} \end{array}$$

*f* is the frequency in Hertz.

The Mel-scale Frequency Cepstral Coefficients (MFCC) is a cepstral parameter extracted in the Mel-scale frequency domain [11]. MFCC were extracted from each clip file as the feature. The MFCC extraction algorithm usually includes windowing the signal into frames, and applying the fast Fourier transform (FFT) on frames to get the short-time Fourier transform spectrum (STFT). Then, the STFT spectrum was filtered with Mel-filter banks to get the Mel-spectrum, the Mel-spectrum was transformed into Mel-frequency cepstrum by taking the logarithm and then followed by applying the discrete cosine transform (DCT) to get MFCC coefficients. The MFCC feature vector describes the power spectral envelope of a single frame.  Figure 3 shows the waveform, the Mel-spectrum, and the MFCC of a snoring sound clip with a duration of 60 seconds.

#### 2.1.3. Similarity Calculation

The MFCC of each clip is a two-dimensional matrix, each column presents for a frame, and each row in the matrix corresponds to the Mel-frequency cepstral coefficients for the corresponding frame. As the respiratory sound signal is quasiperiodic, the MFCC matrix can be averaged by each row to get a one-dimension vector. As a vector can be presented as a point in a high-dimension space by its Cartesian coordinates, the MFCC matrix can be presented as points in a high-dimension space. The distance between the two clips can be measured by the distance between these two points. Based on our experiences, the Euclidean distance gave the most satisfying cluster result. The Euclidean distance between two points in Euclidean space is the length of a line segment between the two points. In general, if *p* and *q* are two points in *n*-dimensional Euclidean space, then the distance between them can be calculated by the following equation:

(3) $$\begin{array}{c} d\left(p,q\right)=\sqrt{{\left(p_{1}-q_{1}\right)}^{2}+{\left(p_{2}-q_{1}\right)}^{2}+\cdots +{\left(p_{n}-q_{n}\right)}^{2}}\text{.} \end{array}$$

#### 2.1.4. Agglomerative Hierarchical Clustering

Hierarchical clustering is a method of cluster analysis that can discover the structure of the dataset in an unsupervised way. It seeks iteratively merging nodes into bigger clusters (agglomerative), or divisive clustering nodes in the inverse (divisive) to build a hierarchy of all data. Agglomerative hierarchical clustering (AHC) is the most common type of hierarchical clustering [12, 13]. Pairs of clusters are successively merged until all clusters have been merged into one big cluster that contains all objects. At each iteration, two nodes or clusters, which have the minimum distance are merged. The result is a tree-based representation of all the objects, named a dendrogram. The number of clusters needs to be set before the algorithm begins.

A 120 minutes length file (2 hours) was selected from all the data and segmented into 60 seconds length clips for demonstration; therefore, 120 clips were used in the experiments. The STFT spectrum window length is 1000 ms with an overlap of 500 ms. The 40 Mel-scale filters were set in MFCC extraction. The distance matrix size is a symmetry matrix with a size of (120, 120). The dendrogram of the clustering result is shown in Figure 4. Based on the structure of the dendrogram, the dendrogram was divided into 3 clusters. Cluster 1, cluster 2, and cluster 3 are presented with cyan, magenta, and yellow, respectively. The dendrogram is shown in Figure 4, and the dendrogram is truncated for showing the main structure for the better visualization effect. The properties of each cluster are listed in Table 1.

One clip was chosen from each cluster as an example for analysis. The waveform and Mel-spectrum of examples present for each example are shown in Figure 5.  Figure 5(a) is a spectrum of snoring. The snoring sounds are almost the same in amplitude and evenly spaced, the pitch of the snoring sound is in the low-frequency range and corresponds to a fundamental frequency with associated harmonics, and inspiratory is louder than expiratory.  Figure 5(b) is a spectrum of normal respiration. It is characterized by a broader spectrum and is audible both during the inspiratory and expiratory phases.  Figure 5(c) is a spectrum of uncertain types. The signal is very weak, and its spectrum has almost equal energy at frequencies below 2000 Hz. It is mixed with the weak breath, but the signal level is insufficient for analysis.

### 2.2. Snoring Classification Based on K-Means Algorithm

Snoring occurs when the upper airways collapse, air moves around the floppy tissue near the back of the throat, and causes the tissue to vibrate. Simple snoring (also called benign snoring) occurs when there is a partial collapse of the soft tissues. As such, simple snoring is generally not considered a health threat. Apneic Snoring (also called obstructive sleep apnea-related snoring) is caused by partial or complete obstruction of the airway, and apneic snoring causes a partial or complete airflow stop, resulting in little or no oxygen going to the blood [14, 15]. For the apneic snoring, at the end of the obstruction, the closed upper airway is suddenly opened, and the pressures of the upper and lower airflows are suddenly balanced, causing the upper airway to repeat multiple openings and closings in a short period, producing a popping sound. The collapse degree and resistance of the upper airway may vary greatly from the beginning to the end of inspiration, thus, affecting the vibration of the upper airway tissue [16]. The snoring sounds in patients with obstructive sleep apnea and with simple snoring have different characteristics and effects on breath quality. It is essential to discriminate between these two different types of snoring for evaluating the influence on tidal volume.

Formant frequencies represent the resonance frequencies of the airways and change with the upper airway anatomy. A formant is the broad spectral maximum produced by an acoustic resonance of the human vocal tract [17]. Formants represent the direct source of pronunciation information, and the extraction and trajectory tracking of formants play an important role in speech recognition and speech synthesis. The formants *F*1–*F*3 are the three lowest resonant frequencies of the vocal tract. *F*1 is associated with the degree of pharyngeal constriction and the height of the tongue. *F*2 reflects the degree of the tongue's relative advancement position to its neutral position. *F*3 is related to the degree of lip rounding. Among *F*1–*F*3, *F*1 carries more information than others as it is associated with severity of apnea. Like speech pronunciation, snoring sounds are also produced depending on the shape and physical conditions of the upper airway, the formant of snoring can be extracted as a snoring feature [18]. Ng et al. proposed that apneic snoring has a high formant frequency than simple snoring in *F*1, and a threshold value of *F*1 = 470 Hz can be used to distinguish apneic snoring from simple snoring [19]. Sola Soler et al. suggested that the formant standard deviation of OSA snoring is higher than simple snoring [20].

These studies used the formant parameters to distinguish simple snoring from apneic snoring, and all emphasized the decisive role of *F*1. However, some cases may be misjudged by these methods. The reason is that the difference between the speech formant and the snoring formant is not considered. The most important formant analysis in speech processing is the formant tracks. The spacing between the word formant is not taken into consideration in speech processing. On the contrary, in applications such as speech recognition, the effect of spacing needs to be eliminated. The frequently used methods are dynamic time warping (DWT). By locally scaling the speech sequence, DWT eliminates the influence of speech rate and word spacing, so that the morphology of the two speech sequences is as consistent as possible, and the maximum possible similarity is obtained. But in snoring recognition, the interval between breathing is an important parameter as it is associated with airflow reduction time, and the interval of apneic snoring is usually larger and more irregular than simple snoring. To solve this problem, this paper extracted the standard deviation of the formant interval, together with the standard deviation of the formant frequencies as parameters, and used the *K*-means algorithm to discriminate between simple snoring and obstructive snoring by unsupervised clustering. *K*-means clustering is an unsupervised learning algorithm, it groups the unlabeled dataset into different clusters [21]. *K* defines the number of predefined clusters that need to be created in the process, here the *K* is set as 2.

The linear predictive analysis (LPC) method is one of the fast and more effective formant frequency estimation methods. The system function of the human vocal tract can be uniquely determined by a set of linear prediction coefficients, so the effect of vocal tract modulation can be estimated through LPC analysis. The formant of snoring can be obtained. The sound signals were windowed with a Hamming window of 20 ms with 50% overlap. In each window, a 14th-order LPC analysis is performed, and the LPC parameters were calculated via the Yule–Walker autoregressive method with the Levinson–Drubin recursive procedure. The standard deviation of *F*1 frequencies and the standard deviation of F1 interval are extracted to form a 2-dimensional feature vector. The snoring cluster result is shown in Figure 6. The apneic snoring and simple snoring are marked with red and cyan dots, respectively. After *K*-means clustering, the snoring cluster result of AHC is divided into 2 subclusters: cluster 0 and cluster 1. The property of all 4 clusters is shown in Table 2. The spectrum of the example clip chosen from cluster 0 and cluster 1 is shown in Figure 7, the formant is displayed with black dots on the spectrum.

### 2.3. Tidal Volume Level Estimation

For each cluster, different parameters are extracted and the corresponding tidal volume levels are determined based on these parameters. The tidal volume levels are divided into three grades: high, medium, and low. The tidal volume level is calculated for each cluster.

Cluster 2 contains the normal breathing clips, although there are fluctuations during normal respiration, the tidal volume levels of normal breathing can roughly be set as high.

Cluster 1 contains simple snoring. According to Hoffstein's research, simple snoring does not cause a sustained deterioration of MnO_2_ (mean nocturnal oxygen saturation) but cause significantly the variability of LoO_2_ (lowest nocturnal oxygen saturation) [22]. Based on this research, the tidal volume level during simple snoring beginning is similar to normal respiration, but after a certain duration, the fluctuation of nocturnal oxygen saturation increases and deteriorates ventilation quality at a moderate level. Although the accurate SpO_2_ drop time is not clear, according to the research by Gruber, the interval to equilibration of oxygen saturation is within 4.5 minutes [23]. Therefore, the SpO_2_ drop threshold is set at 4 minutes, meaning that when the normal breathing ends and simple snoring starts, after approximately 4 minutes, the SpO_2_ drops to a medium level with high probability.

Cluster 0 contains apneic snoring. The breathing pause lasts longer than normal breathing during apnea. Based on the research by Ma et al., nocturnal hypoxemia severity is proportional to the pause time [24]. To evaluate the severity of hypoxemia, the maximum breathing pause interval (MBPI) is calculated as a parameter. According to the apnea definition, the threshold to distinguish the low/medium grade of apneic snoring is set to 10 seconds. The criterion for tidal volume level estimation is listed in Table 3.

## 3. Results and Discussion

The SpO_2_ is a reading that shows the amount of oxygen available in human blood to deliver to the heart, brain, lungs, and other muscles and organs. The LoO_2_ (lowest nocturnal oxygen saturation) is the lowest SpO_2_ value during a certain time and has a high correlation with tidal volume. The LoO_2_ is divided into 3 levels: large than 95% is considered a high level, less than 90% is considered low (hypoxemia), and between 95% and 90% is considered medium (mild) hypoxemia. The summarized results are shown in Figure 8. The first row is the clustering result, the *x*-axis represents the clip index, and each clip is 60 seconds in length. Each clip is classified into apneic snoring/simple snoring/breathing/uncertain types. The second row is the tidal volume level calculated by the proposed algorithm. The third row is the LoO_2_, which is divided into high/medium/low levels, and the uncertain level corresponds to the uncertain clustering type. The fourth row is the SpO_2_ level that is used to calculate the third row.

Six clips were selected as representatives, which are shown in Figure 9.  Figure 9(a) is a normal respiration state at the 13th minute, the corresponding SpO_2_ is stable and LoO_2_ is above 95%.  Figure 9(b) is apneic snoring with MBPI ≤ 10 at the 19th minute, the SpO_2_ fluctuates, and LoO_2_ is between 95% and 90%.  Figure 9(c) is apneic snoring with MBPI > 10 at the 20th minute, the SpO_2_ fluctuates dramatically, and LoO_2_ is below 90%.  Figure 9(d) is simple snoring at the 16th minute, the SpO_2_ is at a high level as in (a).  Figure 9(e) is simple snoring at the 43th minute, the SpO_2_ drops slightly, and the LoO_2_ drops to between 95% and 90%.  Figure 9(f) is an uncertain case by which the signal is insufficient to calculate the SpO_2_ level.

The accuracy is calculated by equation (4). Six patients with different apean-hypopnea index (AHI) were selected to test the effectiveness and robustness of the proposed method. AHI is defined as the number of apnea or hypopnea per hour during sleep. It is used as a parameter for the evaluation of the OSA severity. AHI less than 15 is considered mild apnea. AHI between 15 and 30 denotes moderate apnea, while a greater than 30 is considered severe. The characteristic of selected data and algorithm performance are shown in Table 4. The algorithm accuracy is 88.3% in the group with mild apnea. As for the moderate apnea group, the algorithm accuracy slightly drops to 85.8%. In the severe apnea group where the sound signal contains ambient noise, the algorithm accuracy is still above 83%.

(4) $$\begin{array}{c} Accuracy=\frac{correct\;prediction\;number}{total\;number-uncertain\;number}\text{.} \end{array}$$

## 4. Conclusion

In this study, a tidal volume level prediction method is proposed based on unsupervised clustering and snoring parameters. This method can provide a coarse-grained tidal volume level estimation that does not need any calibration. In addition, this method can be used for sleep breathing monitoring in a home environment. However, the accuracy of the method in this study is not very well because noise such as ambient noise will cause misjudgement, also breathing during sleep is affected by many other factors such as sleep position, pulmonary disease, and body movement, these factors cannot be captured by breathing sound. We are going to improve the performance by incorporating other factors in the future.

## Figures and Tables

**Figure 1:** The flow of the proposed method.

**Figure 2:** Data extracted from PSG-audio: (a) SpO_2_; (b) Tracheal sound; (c) Respiratory events.

**Figure 3:** Spectrum of a snoring sound clip. (a) The waveform; (b) the Mel-spectrum; (c) MFCC.

**Figure 4:** The dendrogram of cluster result.

**Figure 5:** The example waveform and Mel-spectrum of each cluster: (a) Example of cluster 1; (b) Example of cluster 2; (c) Example of cluster 3.

**Figure 6:** The apneic snoring/simple snoring cluster result.

**Figure 7:** Example spectrum and formant of; (a) cluster 0 and (b) cluster 1.

**Figure 8:** The prediction result: (a) cluster label, (b) tidal volume level prediction, (c) LoO_2_, and (d) SpO_2_.

**Figure 9:** The representative state in prediction result. (a) Normal respiration; (b) apneic snoring with MBPI ≤ 10; (c) apneic snoring with MBPI > 10; (d) simple snoring with normal SpO_2_; (e) simple snoring with SpO_2_ drops slightly; (f) uncertain signal.

**Table 1:** Characteristics of each cluster.

Cluster no	Property	Clip number
1	Snoring	94
2	Normal respiratory	12
3	Uncertain	14

**Table 2:** Characteristics of after SS/AS classification.

Cluster no	Property	Clip number
0	Apneic snoring (AS)	29
1	Simple snoring (SS)	65
2	Normal respiration	12
3	Uncertain	14

**Table 3:** The criterion for tidal volume calculation.

Cluster no	Property	Criterion	Breathing quality
0	Apneic snoring	MBPI ≤ 10 second	Medium
		MBPI > 10 second	Low

1	Simple snoring	Last time < 4 minutes	High
		Last time ≥ 4 minutes	Medium

2	Normal respiration	All	High

**Table 4:** Algorithm accuracy on data with different characteristics.

Apnea severity	Patient number	Data length (hour)	Data characteristic	Algorithm accuracy (%)
Mild	1	2	Mild apnea, no simple snoring	88.3
Moderate	3	6	Moderate apnea, little simple snoring	85.8
Severe	2	4	Severe apnea, little simple snoring, containing ambient noise	83.3

## Data Availability

The data supporting the current study are available from the corresponding author upon request.
